This article has been retracted.

# Network Pharmacology-Based Study on the Active Component and Mechanism of the Anti-Non-Invasive and Invasive Bladder Urothelial Carcinoma Effects of Zhuling Jisheng Decoction

**DOI:** 10.1155/2021/7667707

**Published:** 2021-12-31

**Authors:** Chenyu Ma, Jianlong Wang, Na Zhao, Zhenya Pan, Yi Lu, Miao Cheng, Min Deng

**Affiliations:** ^1^Third People's Hospital, Ningbo City, Zhejiang Province, No. 51-139, Zhouxi Highway, Cixi, China; ^2^Xi'an International Medical Center Hospital, China; ^3^Emergency Medicine Department, Zhejiang Hospital of Integrated Traditional Chinese and Western Medicine, China; ^4^Yiwu Fuyuan Private Hospital, China; ^5^Department of Oncology, The Third People's Hospital of Hangzhou, Hangzhou, Zhejiang, China

## Abstract

Zhuling Jisheng decoction is employed for the treatment of bladder urothelial cancer in clinical practice of traditional Chinese medicine. However, there are few studies on its precise mechanism. For the antibladder cancer action of Zhuling Jisheng decoction, a network pharmacological technique was used to design a component/target/pathway molecular regulatory network. The TCMSP dataset was used to identify the chemical makeup of Zhuling Jisheng decoction, which was then analyzed and assessed for oral bioavailability and pharmacological similarity. The chemical composition of Zhuling Jisheng decoction was identified through the TCMSP database, and it was evaluated and screened based on oral bioavailability and drug similarity. The GEO database was searched for genes associated with urothelial bladder carcinoma, and gene targets associated with bladder urothelial cancer resistance were chosen by comparison. The function and linked pathways of the target genes were examined and screened using annotation, visualization, and a comprehensive discovery database. The impact of Zhuling Jisheng decoction on urothelial bladder cancer was studied using Cytoscape software to create a component/target/pathway network. Finally, 69 and 55 target genes were discovered for noninvasive bladder urothelial cancer and invasive bladder urothelial cancer, respectively. In noninvasive urothelial cancer, 118 pathways were highly enriched, including the TNF signaling pathway and the IL-17 signaling route. 103 pathways were highly enriched in invasive urothelial cancer, including the p53 signaling route, bladder cancer route, and calcium signaling route. There were 18 and 15 drug targets associated with noninvasive and invasive bladder urothelial carcinoma prognoses. Many signaling pathways directly act on tumours, and indirect pathways inhibit the development of bladder urothelial carcinoma. This research establishes a scientific foundation for further research into the framework of action of Zhuling Jisheng decoction in the therapy of bladder urothelial cancer.

## 1. Introduction

The most frequent malignant tumour in the urinary system is bladder cancer. Each year, more than 470,000 people in the world are diagnosed with bladder cancer for the first time [1]. Furthermore, men are three to four times as likely as women to get bladder cancer [2]. Urothelial cell carcinoma, squamous cell carcinoma, and adenocarcinoma are the most prevalent bladder malignancies, followed by metastatic malignancies, small cell carcinomas, and carcinosarcomas. The most frequent urological malignancy of human bladder cancers, urothelial carcinoma of the bladder, accounts for more than 90% of all bladder cancers, divided into two categories focused on the clinical and morphological characteristics [3]. The majority of urothelial carcinomas constitute noninvasive papillary tumours (PTA stage). These tumours are typically highly differentiated, develop slightly without spreading widely, and have an excellent clinical prognosis, while the remaining one-third of urothelial carcinomas (staged pT1 and above) are invasive tumours with weak differentiation, a rapid rate of progression, and the capacity to metastasize. Bladder cancer has the feature of “three highs:” a high morbidity rate, a high postoperative recurrence rate, and a high fatality rate.

Western medicine relies heavily on surgery to treat bladder cancer, combined with radiotherapy and chemotherapy. But the side effects are considerable, and it is not ideal after healing [4]. Traditional Chinese medicine treatments for cancer show unique advantages in controlling the development of cancer lesions, prolonging the survival time for patients and improving the quality of life. Previous studies have studied the anticancer mechanism of traditional Chinese medicine in five directions: inhibiting cancer cell proliferation, directly killing cancer cells, reducing cancer cell metastasis ability, inducing cancer cell apoptosis, and inhibiting tumour blood vessel formation [5]. For example, Yiqi Jianpi Huaji decoction has the effect of reversing multidrug resistance [6]. In gastric cancer rats, Huayu Jiedu Fang can lower the levels of IL-6, IL-10, and TNF-*α*, as well as the inflammatory response [7]. Weipixiao, a traditional Chinese medicine ingredient, inhibits lung cancer cell angiogenesis by decreasing “hypoxia-inducible factor (HIF-1) and vascular endothelial growth factor (VEGF)” [8]. As a result, traditional Chinese medicine offers a valuable supplement to developing innovative cancer therapies.

Zhuling Jisheng decoction (ZLJSD), a compound prescription for bladder cancer based on traditional Chinese medicine theory, contains *Polyporus umbellatus* (Pers.) Fries, *Astragali Cpmplanatisemen*, *Herba Taxilli*, *Pseudobulbus Cremastrae Seu Pleiones*, and *Hedyotis Diffusa Herba*, which can treat bladder cancer [9]. Resent research shows that *Polyporus umbellatus* contains polysaccharides and steroids. Among them, *Polyporus umbellatus* polysaccharides have effects of antitumour and improve immunity [10]. *Pseudobulbus Cremastrae Seu Pleiones* contains phenanthrene, glycosides, and aromatic compounds, which can be utilized to antitumour, antiangiogenesis, and antihypertensive [11]. *Herba Taxilli* contains flavonoids and volatile oils, which can be used for anti-inflammatory and antitumour effects; lowering blood pressure, blood sugar, and blood lipids; and enhancing memory [12]. *Astragali Cpmplanatisemen* contains chemical components such as flavonoids, triterpenoid saponins, polysaccharides, sterols, organic acids, and smaller elements such as zinc and manganese, which can be utilized to lower blood pressure and improve cellular immune function, anti-inflammatory, anticancer, and antioxidant effects [13]. *Hedyotis Diffusa Herba* mainly includes terpenes, anthraquinones, flavones, sterols, polysaccharides, organic acids, and alkanes, which can have anti-inflammatory, antioxidant, and neuroprotective effects [14]. Although ZLJSD is used clinically for the treatment of bladder cancer but the peculiar medicinal substances and mechanisms are not clear, so, further investigation is required.

The results of the substantial data study include network pharmacology. Network pharmacology's multicomponent, multitarget, and multichannel network constructive thinking is more suited than traditional single-component, single-target thinking for the complex characteristics of the traditional Chinese medicine complex. From a certain point of view, network pharmacology as a new method provides a large amount of information on the pharmacological effects of single-flavour and Chinese compound medicine. It can analyze traditional Chinese medicine recommendations from a modern pharmacological perspective. It can also assist in researching and developing current Chinese drugs and new dosage forms. As a result, integrating different components, different target characteristics, and network pharmacology in traditional Chinese medicine prescription might help researchers better understand the material foundation and mechanism of action in illness therapy [15]. Sun et al. employed network pharmacology technology to identify the active components and signaling pathways in Dachengqi decoction and investigate the molecular framework of DCQD in the therapy of acute pancreatitis. The results show that 17 prompt ingredients of DCQD can be promoted by “regulating the PI3K/AKT signaling pathway” apoptosis and inhibition of pathological damage and inflammation to improve acute pancreatitis [16]. Tang et al. used network pharmacology methods to find “37 potential targets of the Mahuang Fuzi Xixin decoction for treating allergic rhinitis, including drug similarity assessment, oral bioavailability prediction, multiple drug-target predictions, and network analysis of active ingredients and potential targets.” The objective has something to do with allergic rhinitis. In addition, four of the expected components have been discovered as having anti-inflammatory properties [17]. Shi et al. used network pharmacology and validation studies to investigate the method of Danggui Buxue decoction's blood-enriching action for treating blood deficiency syndrome and discovered that it works by increasing immunity and increasing immunity hematopoiesis simultaneously [18]. The studies above demonstrated that network pharmacology has gradually begun to penetrate various aspects of traditional Chinese medicine research, exploring new aspects of traditional Chinese medicine and systematically explaining the component-target relationship and pharmacological mechanism of single and compound traditional Chinese medication. Collecting traditional Chinese medicine ingredients, predicting the target of the action, clarifying the action mechanism of single Chinese medicine, and discovering the latest indications of traditional Chinese medicine have important application value.

The method and molecular targets of ZLJSD in the therapy of bladder urothelial carcinoma were investigated using a network pharmacological approach in this research study. The TCMSP database was used to identify the active chemicals of ZLJSD and their targets. Then, to find bladder urothelial cancer-related sites, we looked at the differently expressed genes among patients with bladder urothelial cancer and healthy people. The likely mechanism of “ZLJSD therapy of BLCA was investigated using gene ontology (GO), Kyoto Encyclopedia of Genes and Genomes (KEGG) pathway analysis, and survival curve.” It will be beneficial to explore the processes of traditional Chinese medicine formulas, uncover pharmacological targets, and serve as a guide for future therapeutic procedures.

## 2. Materials and Methods

### 2.1. Active Ingredient Screening

We utilized the traditional Chinese medicine system's pharmacological databases and analytic platforms (TCMSP, http://lsp.nwu.edu.cn/tcmsp.php) [19] to identify the chemical elements of ZLJSD. This database is used to obtain composition data, such as the composition number, “molecular name, molecular weight, fat-water partition coefficient, number of hydrogen bond donor acceptors, oral bioavailability (OB), intestinal epithelial permeability, blood-brain barrier (BBB), drug similarity (DL), and drug half-life” (HL). We chose to have oral bioavailability (OB) ≥ 30% and drug similarity (DL) ≥ 0.18 [20].

### 2.2. Identify Potential Targets

To discover the matching targets of ZLJSD, these 33 potential compounds were entered towards the DrugBank database (https://www.drugbank.ca/) [21]. After removing 6 compounds that were not linked to any target, 27 were finally selected. A total of 875 targets for 27 compounds were collected.

### 2.3. Targets Related to Bladder Urothelial Cancer

Differentially expressed genes in patients with BLCA are by the GEO databank (https://www.ncbi.nlm.nih.gov/geo/) from series GSE40355 and number of samples: GSM991923-GSM991930 control samples, 8 cases, GSM991931-GSM991938 samples of 8 noninvasive tumour samples (2x pTaG1 and 6x pTaG2), and GSM991939-GSM991946 of 8 invasive samples of tumour (1x pT1G1, 4x pT1G3, and 3x pT2G3). Genes with FDR values < 0.05 and log_2_(fold change) > 1 were regarded to have BLCA linked and differential objectives.

### 2.4. Network Construction

ZLJSD's complicated target network was built and visualized in Cytoscape 3.7.2 software. The STRING database is a database that holds information on direct and indirect protein interactions. For the degree of interaction, each protein is under a *P* value. A higher value leads to more confidence in the interaction of protein. Genes relevant to the therapy of ZLJSD bladder cancer have been uploaded for protein interaction to the online STRING database. Data were selected and imported into the software Cytoscape to generate the PPI network for ZLJSD with a high confidence score of 0.7 detect System-level protein–protein interactions. The core PPI network of ZLJSD's calculated objective and the noninvasive and invasive BLCA targets were shown using the Cytoscape MCODE program.

### 2.5. Bioinformatic Analysis

GO analysis was done utilizing a Database for “Annotation, Visualization, and Integrated Discovery” (DAVID) (https://david.ncifcrf.gov, v6.8) to evaluate the biological function molecular function and cellular component. In the genes (FDR < 0.05), functional categories have been enriched and the top 20 functioning categories of GO have been picked. For pathway analysis alone, DAVID that assigned the Kyoto Encyclopedia of Genes and Genome (KEGG) database was utilized. For subsequent investigation, pathways with significant FDR < 0.05 alterations were discovered [22].

### 2.6. Relationship between Key Target Genes and Patient Prognosis

Prognostic Analysis of the Cancer Genome Atlas (TCGA) is a project NHGRI and NCI cooperation. The TCGA database is an associated project (NCI). TCGA carried out 33 tumours by sequencing. In this work, the BLCA grouping in TCGA analysis analyzes and draws Kaplan-Meier survival curve forecasts in the forecast of noninvasive urothelial cancer and invasive urothelial cancer, which examines the association of important target genes with the forecast.

## 3. Results

### 3.1. Composite Target Network Analysis

The potential compounds were identified for twenty-seven ZLJSD (Table 1). As Figure 1(a) shows, the GE Odds Database, 2485 of which were upregulated and 3104 downregulated, shows 5589 genes related to noninvasive BLCA. As shown in Figure 1(b), 4,460 distinct genes are in invasive BLCA with upregulation of 2173 and downregulation of 22,287 of them. As Figure 1(c) shows, there are 181 distinctive genes, upregulated by 158 and downregulated by 23, for invasive versus noninvasive BLCA. ZLJSD's composition network was built utilizing the tested compounds and their objectives. As shown in Figure 2(a), there were 90 nodes (21 compounds for ZLJSD and 69 compound goals) in the drug and noninvasive-urothelial carcinoma network, as well as 166 borders indicating interactions between compounds. As shown in Figure 2(b), 76 nodes (21 compounds and 55 medicines in ZLJSD) and 147 edges indicate that the compound objective interaction is present in the medication and invasive-urothelial carcinoma network. Within noninvasive & invasive BLCA, the Venn diagram shows 39 intersection targets of ZLJSD (Table 2).

### 3.2. Construction of the PPI Network

To examine the working link between the target genes and the differential genes in BLCA, a PPI network was established utilizing the STRING database and visual synthesis was carried out using Cytoscape. The PPI network was used to examine the possible 69 ZLJSD goal genes for noninvasive BLCA therapy. Results indicated that the connection between protein and function was 90 nodes and 166 edges (Figure 3(a)). The MCODE plug-in confirms the list of working PPI network modules and the relevant significant ones (Figure 3(b)). Module 1 (score: 6000) comprises 6 nodes and 15 edges. The seed gene is PRKCA; module 2 (score: 4.5) is composed of 5 nodes and 9 edges; the seed gene is IL-1*β*; module 3 (score: 4) is composed of 4 nodes and 6 edges, and the seed gene is BIRC5. Module 4 (score 3) consists of 3 nodes and 3 edges, and the seed gene is CHRM2. Module 5 (score 3) consists of 3 nodes and 3 edges, and the seed gene is ADRA1B. Module 6 (score 2.8) consists of 6 nodes and 7 edges, and the seed gene is MMP2. The potential 55 target genes for treatment of invasive-BLCA in ZLJSD, showing 76 nodes and 147 edges (Figure 3(c)), are the interaction between protein and function. The MCODE plug-in is utilized to confirm the list of PPI network functional modules and the corresponding meaningful modules listed (Figure 3(d)). Module 1 (score: 4.444) comprises 10 nodes and 20 edges. The seed gene is CHRM2; module 2 (score: 3.333) consists of 4 nodes and 5 edges, and the seed gene is CDK1.

### 3.3. GO and KEGG Enrichment Analysis

The DAVID pathway boosted analysis was conducted by the GO and KEGG on 69 benchmarks for the recognized noninvasive urothelial carcinoma and 55 targets for invasive urothelial carcinoma. Cellular components and molecular functions for applicant target GO have been assessed based on biological processes. As shown in Figure 4(a), 718 GO conditions in noninvasive urothelial cancer (FDR < 0.05), 620 in biological pathways, 43 in cellular constituents, and 55 in molecule functions were highly enriched. GO keywords that are highly abundant in biological mechanisms in cellular constituents and molecular activities comprise cell proliferation control, organic reaction, endogenous stimulus reaction, and steroid hormone stimulus reaction. Invasive urothelial carcinoma (FDR < 0.05), 483 biological mechanisms, 51 cell components, and 45 molecular activities were highly enriched by 579 GO keywords, as shown in Figure 4(b). In additional Table 1, the data evaluated by GO is displayed. Including cell proliferation, apoptosis regulation programmed mortality control of cells, and organic reaction, these GO keywords are significantly abundant in biologic processes, cell components, and molecular function. Common BP ZLJSD was fortified with 404, 31 for CC, and 38 for MF for the therapy of noninvasive BLCA. The data may be found in Table 2.

During the therapy of BLCA, the KEGG pathway study revealed the pathways that were greatly influenced by ZLJSD. As indicated in Figure 5(a), there have been 118 highly enriched pathways (FDR < 0.05, TNF signal pathway), IL-17 signal route, AGE-RAGE signaling route in diabetic problems, NF-kappa B signaling system, etc. in the therapy and therapy of noninvasive urothelial cancer. Data are given in additional Table 3 for the KEGG pathway analysis. 103 substantially enriched pathways (FDR < 0.05), comprising pathway p53s, bladder cancer, and pathways of calcium signaling, were found as shown in Figure 5(b) for the therapy of invasive urothelial carcinoma. Data are included in additional Table 3 for KEGG pathway analysis. 93 frequent approaches of treating noninvasive and invasive BLCAs for KEGG are enhanced.

### 3.4. Genetic Pathway Network Analysis

A network of gene pathways was built on a very rich network and genes that control these pathways, as shown in Figure 6. The BC noninvasive urothelial carcinoma topological study of 20 pathways and 34 genes was carried out. Green is the destination gene, while pink is the network path. The most extensive core goal gene has been found in Figure 6(a). Invasive urothelial cell carcinoma topological analysis using BC was carried out in 20 pathways and 41 genes, as shown in Figure 6(b). The target gene is blue, and the network route is yellow. The diagram in the network demonstrates that IL-6 has the greatest core gene. They might be a significant BLCA ZLJSD target.

### 3.5. Prognostic Analysis of ZLJSD Targets

The TCGA database contains expression and clinical data for 33 tumours. Prognostic analysis using the TCGA database to explore the impact of core genes on the prognosis of BLCA found that survival analysis of noninvasive urothelial carcinoma showed that 18 targets are associated with prognostic survival as shown in Figure 7; the overall survival of patients with high gene expression and those with lower than low expression include ADRA1D, ADRA1A, CALM1, CHRM2, COL3A1, CYP1B1, DPP4, GJA1, JUN, MAOB, PGR, PTGER3, PTGS1, RUNX1T1, and SLC2A4. The general survival of high-gene activity patients is greater than of low expression, including PPARG and TNFSF15. The analysis of survival of invasive urothelial cancer is shown in Figure 8. There have fifteen targets related to prognostic survival. The general survival of high-gene activity patients is lower than those with low expression, ACACA, ADRA1D, ADRA2A, CALM1, CHRM2, CYP1B1, JUN, MAOB, PGR, PTGER3, PTGS1, RUNX1T1, and SLC2A4; the overall survival of patients with high gene expression is higher than those with low expression, including PPARG and VEGFA. The variation (logrank *P* < 0.05) was significant statistically. The findings of the examination of other genes were not significant statistically.

## 4. Discussion

We discovered that ZLJSD could significantly improve the symptoms of bladder cancer patients, and we believe that this is due to its antibladder cancer activity. As a result, we use network pharmacological approaches to investigate probable processes.

We employed oral bioavailability (OB) of 30 percent and drug similarity (DL) of 0.18 to find 21 substances with disease targets: “beta-sitosterol, quercetin, kaempferol, and stigmasterol,” as per the herb-disease network. Beta-sitosterol, for example, efficiently reduces tumour cell development by decreasing proliferation and has antibladder cancer effects [23]. Kaempferol is a flavonoid that suppresses bladder cancer cell development via the c-Met/p38 signaling pathway, hence preventing bladder cancer development, invasion, and metastasis [24].Quercetin, is a flavonoid, a kind of polyphenolic substance that suppresses bladder cancer cell proliferation, cell proliferation, and hypermethylation. The decrease of mutant P53 and survivin proteins may be connected to quercetin-induced apoptosis [25]. In a nutshell, these active components form the foundation for ZLJSD's potential anticancer action on bladder cancers.

We used the target-pathway network, together with the findings of the GO analysis, to hypothesize that the probable strategy of bladder cancer treatment by ZLJSD is connected to biological functions such as inflammatory response, proliferation, angiogenesis, apoptosis, and cell senescence.

### 4.1. Cell Proliferation

Aberrant cell proliferation is a crucial feature of malignancies. The interphase and mitosis of the preparatory phase should be carried out by cell growth and separation. Currently, the overexpression of cyclin and the loss of cyclin-dependent kinase (CKI) inhibitors in the stage are frequently associated with cell malignancy. Cyclin-related kinase 1 (CDK1) is a protein kinase in serines/threonines that plays a vital function in the cell proliferation regulation at a G2/M cell-cycle stage. The required prerequisite for all eukaryotic cells to divide has been taken into consideration till now. CDK1 inactivation of CDK1 causes mitosis to cease [26]. CCNB1 has been acknowledged as a useful screening tool in diagnosing patients with a high recurrence probability and intravesical reaction who are nonmuscular invasive bladder cancer [27]. Downregulation of DNA reparation-related checkpoint protein kinase 2 (CHEK2) is associated with poor prognostic for certain cancers. Studies on the CHEK2 involvement in BLCA have shown that a decrease of CHEK2 expression is an independent progression predictor and an inadequate progressive disease-free survival [28]. CDK1 inhibition of the expression by quercetin and kaempferol may lead to the action of zLJSD on cell proliferation, which further regulates the signaling pathway of the cell cycle. Quercetin can proactively influence DNA repair through CCNB1, CHEK2, and cell cycle effects. Furthermore, quercetin can modulate MAPK via PRKCB and FOS to regulate cell proliferation more.

### 4.2. Apoptosis

The suppression of apoptosis plays an essential part in the genesis and progression of malignancies in increased cell proliferation [29]. Another of the important aspects of apoptosis is the production and regulation of the BCL-2 family. The BCL-2 is an apoptosis protein inhibitor, a PI3K-AKT signal route, and a signal route for the P53 apoptosis regulator [30, 31]. In ZLJSD, beta-sitosterol, quercetin, and kaempferol are substances that operate on BCL-2. In addition, in the CASP cascade, the direct regulation of CASP8 and CASP3 by beta-sitosterol, quercetin, and kaempferol may be an essential component of ZLJSD in regulating apoptosis [32].

### 4.3. Inflammation

Stimulation of inflammatory reactions can lead to the release of tumours into an inflammatory microenvironment of many elements which support their proliferation [33]. TNF is an inflammatory factor that is influential. It can contribute not just to apoptosis but also to cell survival and growth signals. In the inflammatory response [34], NF-*β*B is a crucial factor. The apoptosis protein BCL-2 not only may access the nucleus and speed up the subsequent development of inflammatory molecules like IL-1B, IL-6, and PTGS2 but also prevent apoptosis. Quercetin and kaempferol components in ZLJSD can impact the overall inflammatory reaction through inhibitors of RELA upstream expression [35, 36]. The NF-ŢB signaling route and the IL-6 downregulated route may be implicated. IL-1B suppresses NF-ŢB release either indirectly or directly and suppresses the production of inflammatory downstream proteins. Three-six-six. Research demonstrates that the participation of specific inflammatory variables has a tight relation between cancer pains [37]. The pain reduction given by ZLJSD bladder cancer tumours can also be linked to its anti-inflammatory activity, accordingly.

### 4.4. Angiogenesis

Angiogenesis depends on tumour development and metastasis [38]. The tumour microenvironment (TME) has a basic property of hypoxia and can activate the HIF hypoxia gene transcription triggering the proangiogenic factor VEGF production [39]. VEGF is an important proangiogenic factor. When utilized in conjunction with VEGFR, many downstream signal molecules like PLC-*α* may be activated. PKC, PI3K, MAPK, etc., as well as a signal, may eventually be transmitted towards the cell nucleus and hence achieve the biological impact of VEGF [40]. Quercetin in ZLJSD may affect the expression levels of PTGS2, PRKCA, and PRKCB in the VEGF pathway by acting on HIF1A, VEGFA, and the expression levels of 2 - methoxy-3 - methyl-9,10 - anthraquinone, stigmasterol, and *β*-sitosterol. The expression of quercetin PPP3CA reduces angiogenesis and thus exerts anti-cancer effect.

### 4.5. Cell Senescence

Cell senescence is an irreversible stopping cell cycle system that reacts to several types of cellular stress [41]. Cell ageing can be evident as a significant process for countering cancer. During signal transmission inside the cell senescence signalization pathway, CHEK1 and CHEK2 are essential kinases. It can activate p53 phosphorylation in numerous locations and let p53 trigger cell cycle arrest via downstream target transcript [42]. Four-one-four-one senescence-related cells, known as the senescence-secreted phenotype, release cytokines, chemokines, extra cell matrix protease, and growth factors (SASP). “NF-*κ*B and C/EBP*β*” regulate mainly SASP through direct modulation of the primary inflammation producing SASP regulators (such as IL-6 and IL-8). Secreted SASP factors can improve stability by providing immune system signals and immune recruitment. For instance, “plasminographic activator 1 (PAI1), interleukin 6 (IL-6), interleukin 8 (IL-8), insulin-like growth factor binding protein7,” cell cycle arrests, carcinogenesis (IGFBP7), and growth factor-*β* (TGF-*β*) transformation can lead to cancer cell apoptosis [43]. Secreted SASP also promotes carcinogenesis by generating VEGF or increasing angiogenesis through induction of epithelial transition from one malignancy to another [44]. Therefore, it is necessary to design more potential ageing therapies for a clearly defined method of SASP components. The active components in “formonetin, calycosin, and kaempferide ZLJSD” may operate on the cellular senescence pathway and suppress carcinogenesis using CHEK1, quercetin, CHEK2, RELA, etc.

## 5. Conclusion

Our research predicts the objective of the composition of the ZLJSD by the network pharmacology approach and analyzes its possible anti-BLCA effect mechanism. This approach may address four aspects: antagonizes the systemic inflammatory response and inhibits angiogenesis by decreasing anomalous cell growth and boosting apoptosis. We possess a reason to believe that their anticancer mechanisms for bladder tumours are the indirect or direct synergy between efforts on many multipurpose and several different paths. Further testing, however, is crucial to expose the impact of ZLJSD on antibladder cancer.

## Figures and Tables

**Figure 1:** Heat map of the distinctly expressed genes. The color dots reflect the genes expressed substantially. Red represents upregulated genes and blue represents downregulated genes. (a) Normal samples with noninvasive BLCA, (b) normal samples with invasive BLCA, and (c) invasive sample with noninvasive BLCA sample.

**Figure 2:** Construction of the candidate-target network for ZLJSD against BLCA. (a) ZLJSD treatment of noninvasive BLCA and (b) ZLJSD treatment invasive BLCA. The pink represents targets; the yellow, blue, gray, purple, green, and rose-red represent the compounds from *Astragali Cpmplanatisemen*, *Polyporus Umbellatus* (Pers) Fr., multiple drugs, *Hedyotis Diffusa Herba*, *Herba Taxilli*, and *Pseudobulbus Cremastrae Seu Pleiones*, respectively.

**Figure 3:** PPI network analysis of the potential ZLJSD target genes for BLCA therapy. (a) Demonstrates the target protein PPI network of ZLJSD in noninvasive BLCA targets. (b) Illustrates the analysis of MCODE just after the construction of the ZLJSD target protein PPI while (c) illustrates the ZLJSD invasive BLCA PPI network target protein. (d) Illustrates the MCODE test after the ZLJSD target protein PPI has been constructed.

**Figure 4:** Gene ontology terms for potential ZLJSD targets against BLCA. The top eight GO functional categories were chosen, with an FDR of 0.05 (a) in the noninvasive BLCA, (b) in the invasive BLCA, BP for the biological process, (c) for cellular component, MF for molecular function.

**Figure 5:** Enrichment of putative ZLJSD targets with BLCA by the KEGG pathway. Pathways have been found that have substantial alterations in FDR < 0.05. The spot size is the frequency of genes as well as the color is FDR, (a) in BLCA and (b) in noninvasive BLCA.

**Figure 6:** ZLJSD gene-pathway network against BLCA. (a) In noninvasive BLCA, a topological study of 20 pathways and 34 genes was performed using betweenness centrality. Target genes are shown by blue ellipses, and pathways are represented by green ellipses. (b) Invasive BLCA performed a topological study of 20 pathways and 41 genes using betweenness centrality. The pink ellipses reflect pathways, whereas the green ellipses indicate target genes. The higher the size, the greater the centrality betweenness.

**Figure 7:** 18 drug targets are associated with prognosis in noninvasive urothelial cancer.

**Figure 8:** 15 drug targets associated with prognosis in invasive urothelial cancer.

**Table 1:** The main chemicals in compound ZLJSD.

Medical herbs	Mol ID	Compounds	MW	Structures	Composition
Baihuasheshecao (*Hedyotis Diffusa Herba*)	MOL001659	Poriferasterol	412.69		C_29_H_48_O
Baihuasheshecao (*Hedyotis Diffusa Herba*)	MOL001670	2-Methoxy-3-methyl-9,10-anthraquinoe	252.28		C_16_H_12_O_3_
Baihuasheshecao (*Hedyotis Diffusa Herba*)	MOL000449	Stigmasterol	412.69		C_29_H_48_O
Baihuasheshecao (*Hedyotis Diffusa Herba*)	MOL000358	Beta-sitosterol	414.71		C_29_H_50_O
Baihuasheshecao (*Hedyotis Diffusa Herba*)	MOL000098	Quercetin	302.24		C_15_H_10_O_7_
Sangjisheng (*Herba Taxilli*)	MOL000359	Sitosterol	414.71		C_29_H_50_O
Shancigu (*Pseudobulbus Cremastrae* Seu Pleiones)	MOL000098	Quercetin	302.24		C_15_H_10_O_7_
Shancigu (*Pseudobulbus Cremastrae* Seu Pleiones)	MOL000358	Beta-sitosterol	414.71		C_29_H_50_O
Shancigu (*Pseudobulbus Cremastrae* Seu Pleiones)	MOL000449	Stigmasterol	412.69		C_29_H_48_O
Shancigu (*Pseudobulbus Cremastrae* Seu Pleiones)	MOL007991	2-Methoxy-9,10-dihydrophenanthrene-4,5-diol	242.09		C_15_H_14_O_3_
Shayuanzi (*Astragali Cpmplanatisemen*)	MOL000184	NSC63551	412.69		C_29_H_48_O
Shayuanzi (*Astragali Cpmplanatisemen*)	MOL000358	Beta-sitosterol	414.71		C_29_H_50_O
Shayuanzi (*Astragali Cpmplanatisemen*)	MOL000392	Formononetin	268.27		C_16_H_12_O_4_
Shayuanzi (*Astragali Cpmplanatisemen*)	MOL000417	Calycosin	284.26		C_16_H_12_O_5_
Shayuanzi (*Astragali Cpmplanatisemen*)	MOL004564	Kaempferia	300.26		C_16_H1_2_O_6_
Shayuanzi (*Astragali Cpmplanatisemen*)	MOL009278	Laricitrin	332.263		C_16_H_12_O_8_
Shayuanzi (*Astragali Cpmplanatisemen*)	MOL009289	Calycosin-7-O-beta-D-glucopyranoside	446.41		C_22_H_22_O_10_
Shayuanzi (*Astragali Cpmplanatisemen*)	MOL000098	Quercetin	302.24		C_15_H_10_O_7_
Zhuling (*Polyporus Umbellatus* (Pers) Fr.)	MOL000279	Cerevisterol	430.66		C_28_H_46_O_3_
Zhuling (*Polyporus Umbellatus* (Pers) Fr.)	MOL000282	Ergosta-7,22E-dien-3beta-ol	398.66		C_28_H_46_O
Zhuling (*Polyporus Umbellatus* (Pers) Fr.)	MOL000797	(22e,24r)-Ergosta-7,22-dien-3-one	396.72		C_30_H_30_O
Zhuling (*Polyporus Umbellatus* (Pers) Fr.)	MOL000798	Ergosta-7,22-diene-3*β*-ol	398.66		C_28_H_46_O
Zhuling (*Polyporus Umbellatus* (Pers) Fr.)	MOL000816	Ergosta-7,22-dien-3-one	396.66		C_28_H_44_O
Zhuling (*Polyporus Umbellatus* (Pers) Fr.)	MOL000817	Ergosta-5,7,22-trien-3-ol	396.66		C_28_H_44_O
Zhuling (*Polyporus Umbellatus* (Pers) Fr.)	MOL000822	Polyporusterone G	458.68		C_29_H_46_O_4_

MW: molecular weight.

**Table 2:** Targets of ZLJSD in noninvasive and invasive bladder urothelial carcinoma.

Names	Total	Elements
Invasive BLCA & noninvasive BLCA	39	PTGER3, MMP2, CDK1, FOS, PRKCB, NR3C2, RXRA, PPARG, PTGS1, F3, CHEK2, BCL2, CCL2, PRKCA, SLC2A4, IL-6, PTGS2, BIRC5, PPP3CA, TP63, CCNB1, ADRA2A, CYP1B1, CXCL2, F7, ADH1C, KCNH2, CHRM3, ADRA1D, CAV1, JUN, PGR, CHRM2, RUNX1T1, CCNA2, CASP8, ERBB3, CALM1, and MAOB
Noninvasive BLCA	30	CYP1A2, PPARD, NFKBIA, IGFBP3, CHUK, COL3A1, IGF2, RELA, VCAM1, COL1A1, CYP3A4, TNFSF15, SCN5A, PLAT, SLPI, NCF1, SLC6A4, IKBKB, DPP4, HAS2, MMP3, IL-1B, ICAM1, SELE, IRF1, SOD1, ODC1, PCOLCE, ADRA1B, and GJA1
Invasive BLCA	16	IL-4, CHEK1, ACACA, EIF6, MMP1, STAT1, PSMD3, ADRB2, VEGFA, TOP2A, CDK2, AHR, CASP3, E2F1, E2F2, and ERBB2

**Table 3:** KEGG pathway analysis. 93 frequent approaches of treating noninvasive and invasive BLCAs for KEGG are enhanced.

ID	Description	Gene ratio	Bg ratio	*P* value	*P*.adjust	*q* value	Gene ID	Count
hsa05161	Hepatitis B	14/54	162/8016	1.74*E* − 12	3.56*E* − 10	1.45*E* − 10	BCL2/JUN/CASP3/CASP8/PRKCA/FOS/IL-6/STAT1/PRKCB/BIRC5/E2F1/E2F2/CDK2/CCNA2	14
hsa04933	AGE-RAGE signaling pathway in diabetic complications	11/54	100/8016	3.99*E* − 11	4.09*E* − 09	1.66*E* − 09	BCL2/JUN/CASP3/PRKCA/VEGFA/MMP2/IL-6/STAT1/F3/CCL2/PRKCB	11
hsa05167	Kaposi sarcoma-associated herpes virus infection	13/54	186/8016	1.79*E* − 10	1.23*E* − 08	4.97*E* − 09	PTGS2/JUN/CASP3/CASP8/VEGFA/FOS/IL-6/STAT1/CXCL2/E2F1/E2F2/CALM1/PPP3CA	13
hsa04657	IL-17 signaling pathway	10/54	94/8016	4.73*E* − 10	2.42*E* − 08	9.83*E* − 09	PTGS2/JUN/CASP3/CASP8/FOS/IL-6/MMP1/CCL2/CXCL2/IL-4	10
hsa05163	Human cytomegalovirus infection	13/54	225/8016	1.90*E* − 09	7.80*E* − 08	3.16*E* − 08	PTGS2/CASP3/CASP8/PRKCA/VEGFA/IL-6/CCL2/PTGER3/PRKCB/E2F1/E2F2/CALM1/PPP3CA	13
hsa04218	Cellular senescence	11/54	160/8016	6.48*E* − 09	2.22*E* − 07	8.99*E* − 08	IL-6/CDK1/CCNB1/CHEK2/E2F1/E2F2/CDK2/CCNA2/CHEK1/CALM1/PPP3CA	11
hsa05170	Human immunodeficiency virus 1 infection	12/54	212/8016	1.11*E* − 08	3.24*E* − 07	1.32*E* − 07	BCL2/JUN/CASP3/CASP8/PRKCA/FOS/CDK1/PRKCB/CCNB1/CHEK1/CALM1/PPP3CA	12
hsa04115	p53 signaling pathway	8/54	72/8016	2.13*E* − 08	5.46*E* − 07	2.21*E* − 07	BCL2/CASP3/CASP8/CDK1/CCNB1/CHEK2/CDK2/CHEK1	8
hsa04020	Calcium signaling pathway	11/54	193/8016	4.60*E* − 08	1.05*E* − 06	4.25*E* − 07	CHRM3/CHRM2/ADRB2/ADRA1D/PRKCA/ERBB2/PTGER3/PRKCB/ERBB3/CALM1/PPP3CA	11
hsa05169	Epstein-Barr virus infection	11/54	201/8016	6.99*E* − 08	1.43*E* − 06	5.81*E* − 07	BCL2/JUN/CASP3/CASP8/IL-6/STAT1/PSMD3/E2F1/E2F2/CDK2/CCNA2	11
hsa05219	Bladder cancer	6/54	41/8016	2.64*E* − 07	4.91*E* − 06	1.99*E* − 06	VEGFA/MMP2/MMP1/ERBB2/E2F1/E2F2	6
hsa05031	Amphetamine addiction	7/54	69/8016	3.30*E* − 07	5.64*E* − 06	2.29*E* − 06	MAOB/JUN/PRKCA/FOS/PRKCB/CALM1/PPP3CA	7
hsa04659	Th17 cell differentiation	8/54	107/8016	4.84*E* − 07	7.64*E* − 06	3.10*E* − 06	RXRA/JUN/FOS/IL-6/STAT1/AHR/IL-4/PPP3CA	8
hsa04668	TNF signaling pathway	8/54	112/8016	6.89*E* − 07	9.85*E* − 06	3.99*E* − 06	PTGS2/JUN/CASP3/CASP8/FOS/IL-6/CCL2/CXCL2	8
hsa05206	MicroRNAs in cancer	12/54	310/8016	7.21*E* − 07	9.85*E* − 06	3.99*E* − 06	PTGS2/BCL2/CASP3/PRKCA/VEGFA/TP63/ERBB2/PRKCB/CYP1B1/E2F1/E2F2/ERBB3	12
hsa01521	EGFR tyrosine kinase inhibitor resistance	7/54	79/8016	8.42*E* − 07	1.08*E* − 05	4.37*E* − 06	BCL2/PRKCA/VEGFA/IL-6/ERBB2/PRKCB/ERBB3	7
hsa04110	Cell cycle	8/54	124/8016	1.50*E* − 06	1.80*E* − 05	7.28*E* − 06	CDK1/CCNB1/CHEK2/E2F1/E2F2/CDK2/CCNA2/CHEK1	8
hsa05166	Human T-cell leukemia virus 1 infection	10/54	219/8016	1.58*E* − 06	1.80*E* − 05	7.28*E* − 06	JUN/FOS/IL-6/CHEK2/E2F1/E2F2/CDK2/CCNA2/CHEK1/PPP3CA	10
hsa05222	Small cell lung cancer	7/54	92/8016	2.38*E* − 06	2.57*E* − 05	1.04*E* − 05	PTGS2/RXRA/BCL2/CASP3/E2F1/E2F2/CDK2	7
hsa05323	Rheumatoid arthritis	7/54	93/8016	2.56*E* − 06	2.62*E* − 05	1.06*E* − 05	JUN/VEGFA/FOS/IL-6/MMP1/CCL2/CXCL2	7
hsa05162	Measles	8/54	138/8016	3.36*E* − 06	3.28*E* − 05	1.33*E* − 05	BCL2/JUN/CASP3/CASP8/FOS/IL-6/STAT1/CDK2	8
hsa01522	Endocrine resistance	7/54	98/8016	3.64*E* − 06	3.39*E* − 05	1.38*E* − 05	BCL2/JUN/FOS/MMP2/ERBB2/E2F1/E2F2	7
hsa05223	Non-small cell lung cancer	6/54	66/8016	4.68*E* − 06	4.18*E* − 05	1.69*E* − 05	RXRA/PRKCA/ERBB2/PRKCB/E2F1/E2F2	6
hsa04625	C-type lectin receptor signaling pathway	7/54	104/8016	5.42*E* − 06	4.63*E* − 05	1.88*E* − 05	PTGS2/JUN/CASP8/IL-6/STAT1/CALM1/PPP3CA	7
hsa01524	Platinum drug resistance	6/54	73/8016	8.47*E* − 06	6.94*E* − 05	2.82*E* − 05	BCL2/CASP3/CASP8/ERBB2/BIRC5/TOP2A	6
hsa05140	Leishmaniasis	6/54	77/8016	1.16*E* − 05	9.11*E* − 05	3.69*E* − 05	PTGS2/JUN/FOS/STAT1/PRKCB/IL-4	6
hsa04970	Salivary secretion	6/54	90/8016	2.84*E* − 05	0.000215397	8.74*E* − 05	CHRM3/ADRB2/ADRA1D/PRKCA/PRKCB/CALM1	6
hsa04370	VEGF signaling pathway	5/54	59/8016	4.36*E* − 05	0.000319433	0.000129578	PTGS2/PRKCA/VEGFA/PRKCB/PPP3CA	5
hsa04215	Apoptosis—multiple species	4/54	32/8016	5.75*E* − 05	0.000398847	0.000161792	BCL2/CASP3/CASP8/BIRC5	4
hsa05205	Proteoglycans in cancer	8/54	204/8016	5.84*E* − 05	0.000398847	0.000161792	CASP3/PRKCA/VEGFA/MMP2/ERBB2/CAV1/PRKCB/ERBB3	8
hsa04921	Oxytocin signaling pathway	7/54	153/8016	6.71*E* − 05	0.000444038	0.000180123	PTGS2/JUN/PRKCA/FOS/PRKCB/CALM1/PPP3CA	7
hsa05160	Hepatitis C	7/54	155/8016	7.29*E* − 05	0.00046711	0.000189483	RXRA/CASP3/CASP8/STAT1/E2F1/E2F2/CDK2	7
hsa04066	HIF-1 signaling pathway	6/54	109/8016	8.37*E* − 05	0.000519791	0.000210852	BCL2/PRKCA/VEGFA/IL-6/ERBB2/PRKCB	6
hsa04725	Cholinergic synapse	6/54	112/8016	9.73*E* − 05	0.000586899	0.000238075	CHRM3/CHRM2/BCL2/PRKCA/FOS/PRKCB	6
hsa04151	PI3K-Akt signaling pathway	10/54	354/8016	0.000104478	0.000611944	0.000248234	RXRA/CHRM2/BCL2/PRKCA/VEGFA/IL-6/ERBB2/ERBB3/CDK2/IL-4	10
hsa04726	Serotonergic synapse	6/54	115/8016	0.000112728	0.000641922	0.000260395	PTGS1/PTGS2/MAOB/CASP3/PRKCA/PRKCB	6
hsa05164	Influenza A	7/54	170/8016	0.000130414	0.000722567	0.000293108	CASP3/CASP8/PRKCA/IL-6/STAT1/CCL2/PRKCB	7
hsa04010	MAPK signaling pathway	9/54	295/8016	0.000135506	0.00072873	0.000295608	JUN/CASP3/PRKCA/VEGFA/FOS/ERBB2/PRKCB/ERBB3/PPP3CA	9
hsa05214	Glioma	5/54	75/8016	0.000138636	0.00072873	0.000295608	PRKCA/PRKCB/E2F1/E2F2/CALM1	5
hsa05133	Pertussis	5/54	76/8016	0.000147646	0.000738228	0.000299461	JUN/CASP3/FOS/IL-6/CALM1	5
hsa05212	Pancreatic cancer	5/54	76/8016	0.000147646	0.000738228	0.000299461	VEGFA/STAT1/ERBB2/E2F1/E2F2	5
hsa05152	Tuberculosis	7/54	180/8016	0.000186086	0.000908277	0.000368441	BCL2/CASP3/CASP8/IL-6/STAT1/CALM1/PPP3CA	7
hsa04621	NOD-like receptor signaling pathway	7/54	181/8016	0.000192575	0.00091809	0.000372422	BCL2/JUN/CASP8/IL-6/STAT1/CCL2/CXCL2	7
hsa04114	Oocyte meiosis	6/54	128/8016	0.000203229	0.000946864	0.000384094	PGR/CDK1/CCNB1/CDK2/CALM1/PPP3CA	6
hsa04926	Relaxin signaling pathway	6/54	129/8016	0.000212049	0.000966002	0.000391857	JUN/PRKCA/VEGFA/FOS/MMP2/MMP1	6
hsa04728	Dopaminergic synapse	6/54	132/8016	0.000240337	0.001071065	0.000434476	MAOB/PRKCA/FOS/PRKCB/CALM1/PPP3CA	6
hsa04012	ErbB signaling pathway	5/54	85/8016	0.000250398	0.001092162	0.000443034	JUN/PRKCA/ERBB2/PRKCB/ERBB3	5
hsa05210	Colorectal cancer	5/54	86/8016	0.000264505	0.001129656	0.000458243	BCL2/JUN/CASP3/FOS/BIRC5	5
hsa04210	Apoptosis	6/54	136/8016	0.000282596	0.001182288	0.000479593	BCL2/JUN/CASP3/CASP8/FOS/BIRC5	6
hsa04915	Estrogen signaling pathway	6/54	138/8016	0.00030581	0.001253821	0.00050861	PGR/BCL2/JUN/FOS/MMP2/CALM1	6
hsa04510	Focal adhesion	7/54	199/8016	0.000344429	0.001384471	0.000561608	BCL2/JUN/PRKCA/VEGFA/ERBB2/CAV1/PRKCB	7
hsa04658	Th1 and Th2 cell differentiation	5/54	92/8016	0.000362266	0.001415656	0.000574258	JUN/FOS/STAT1/IL-4/PPP3CA	5
hsa05203	Viral carcinogenesis	7/54	201/8016	0.000365999	0.001415656	0.000574258	JUN/CASP3/CASP8/CDK1/CDK2/CCNA2/CHEK1	7
hsa04912	GnRH signaling pathway	5/54	93/8016	0.000380906	0.001446032	0.000586581	JUN/PRKCA/MMP2/PRKCB/CALM1	5
hsa05224	Breast cancer	6/54	147/8016	0.000429481	0.001600791	0.000649358	PGR/JUN/FOS/ERBB2/E2F1/E2F2	6
hsa05226	Gastric cancer	6/54	149/8016	0.000461636	0.001664529	0.000675213	RXRA/BCL2/ERBB2/E2F1/E2F2/CDK2	6
hsa05215	Prostate cancer	5/54	97/8016	0.00046282	0.001664529	0.000675213	BCL2/ERBB2/E2F1/E2F2/CDK2	5
hsa04923	Regulation of lipolysis in adipocytes	4/54	55/8016	0.000486421	0.001719247	0.000697409	PTGS1/PTGS2/ADRB2/PTGER3	4
hsa04914	Progesterone-mediated oocyte maturation	5/54	99/8016	0.000508446	0.001766634	0.000716632	PGR/CDK1/CCNB1/CDK2/CCNA2	5
hsa05134	Legionellosis	4/54	57/8016	0.000557794	0.001905798	0.000773083	CASP3/CASP8/IL-6/CXCL2	4
hsa05142	Chagas disease (American trypanosomiasis)	5/54	102/8016	0.00058314	0.001928126	0.000782141	JUN/CASP8/FOS/IL-6/CCL2	5
hsa05146	Amoebiasis	5/54	102/8016	0.00058314	0.001928126	0.000782141	CASP3/PRKCA/IL-6/PRKCB/CXCL2	5
hsa04620	Toll-like receptor signaling pathway	5/54	104/8016	0.000637332	0.002073857	0.000841257	JUN/CASP8/FOS/IL-6/STAT1	5
hsa04928	Parathyroid hormone synthesis, secretion, and action	5/54	106/8016	0.000695221	0.00222688	0.00090333	RXRA/BCL2/PRKCA/FOS/PRKCB	5
hsa05321	Inflammatory bowel disease (IBD)	4/54	65/8016	0.000918763	0.002897638	0.001175422	JUN/IL-6/STAT1/IL-4	4
hsa04720	Long-term potentiation	4/54	67/8016	0.001029849	0.003198774	0.001297577	PRKCA/PRKCB/CALM1/PPP3CA	4
hsa05165	Human papillomavirus infection	8/54	330/8016	0.001505195	0.004605448	0.001868192	PTGS2/CASP3/CASP8/VEGFA/STAT1/E2F1/CDK2/CCNA2	8
hsa04971	Gastric acid secretion	4/54	75/8016	0.001569477	0.00473151	0.001919329	CHRM3/PRKCA/PRKCB/CALM1	4
hsa04380	Osteoclast differentiation	5/54	128/8016	0.001623043	0.004822084	0.00195607	JUN/PPARG/FOS/STAT1/PPP3CA	5
hsa04960	Aldosterone-regulated sodium reabsorption	3/54	37/8016	0.00190982	0.005514268	0.002236853	NR3C2/PRKCA/PRKCB	3
hsa05143	African trypanosomiasis	3/54	37/8016	0.00190982	0.005514268	0.002236853	PRKCA/IL-6/PRKCB	3
hsa04662	B cell receptor signaling pathway	4/54	82/8016	0.002181418	0.006210983	0.002519474	JUN/FOS/PRKCB/PPP3CA	4
hsa05235	PD-L1 expression and PD-1 checkpoint pathway in cancer	4/54	89/8016	0.002941331	0.008259901	0.003350615	JUN/FOS/STAT1/PPP3CA	4
hsa05132	Salmonella infection	6/54	214/8016	0.002993412	0.008292561	0.003363863	BCL2/JUN/CASP3/CASP8/FOS/IL-6	6
hsa04024	cAMP signaling pathway	6/54	216/8016	0.003134975	0.008396427	0.003405996	CHRM2/ADRB2/JUN/FOS/PTGER3/CALM1	6
hsa04261	Adrenergic signaling in cardiomyocytes	5/54	149/8016	0.00315378	0.008396427	0.003405996	ADRB2/ADRA1D/BCL2/PRKCA/CALM1	5
hsa04932	Nonalcoholic fatty liver disease (NAFLD)	5/54	149/8016	0.00315378	0.008396427	0.003405996	RXRA/JUN/CASP3/CASP8/IL-6	5
hsa04713	Circadian entrainment	4/54	97/8016	0.004011834	0.010543923	0.004277124	PRKCA/FOS/PRKCB/CALM1	4
hsa05231	Choline metabolism in cancer	4/54	98/8016	0.004161902	0.010799873	0.00438095	JUN/PRKCA/FOS/PRKCB	4
hsa04064	NF-kappa B signaling pathway	4/54	102/8016	0.004800227	0.012300582	0.00498971	PTGS2/BCL2/PRKCB/CXCL2	4
hsa04022	cGMP-PKG signaling pathway	5/54	167/8016	0.00512959	0.012857065	0.005215446	ADRB2/ADRA1D/ADRA2A/CALM1/PPP3CA	5
hsa04660	T cell receptor signaling pathway	4/54	104/8016	0.005142826	0.012857065	0.005215446	JUN/FOS/IL-4/PPP3CA	4
hsa05014	Amyotrophic lateral sclerosis (ALS)	3/54	57/8016	0.006541874	0.01615764	0.006554319	BCL2/CASP3/PPP3CA	3
hsa05145	Toxoplasmosis	4/54	112/8016	0.006677299	0.016295788	0.006610358	BCL2/CASP3/CASP8/STAT1	4
hsa05202	Transcriptional misregulation in cancer	5/54	186/8016	0.008035734	0.0193803	0.007861585	RXRA/PPARG/IL-6/RUNX1T1/CCNA2	5
hsa04919	Thyroid hormone signaling pathway	4/54	119/8016	0.008247201	0.01943306	0.007882987	RXRA/PRKCA/STAT1/PRKCB	4
hsa04935	Growth hormone synthesis, secretion, and action	4/54	119/8016	0.008247201	0.01943306	0.007882987	PRKCA/FOS/STAT1/PRKCB	4
hsa04152	AMPK signaling pathway	4/54	120/8016	0.0084896	0.019554697	0.007932329	PPARG/ACACA/SLC2A4/CCNA2	4
hsa05135	Yersinia infection	4/54	120/8016	0.0084896	0.019554697	0.007932329	JUN/FOS/IL-6/CCL2	4
hsa04924	Renin secretion	3/54	69/8016	0.011069325	0.025102948	0.010182967	ADRB2/CALM1/PPP3CA	3
hsa05130	Pathogenic Escherichia coli infection	5/54	202/8016	0.011245951	0.025102948	0.010182967	JUN/CASP3/CASP8/FOS/IL-6	5
hsa04068	FoxO signaling pathway	4/54	131/8016	0.011469853	0.025102948	0.010182967	IL-6/CCNB1/SLC2A4/CDK2	4
hsa04650	Natural killer cell-mediated cytotoxicity	4/54	131/8016	0.011469853	0.025102948	0.010182967	CASP3/PRKCA/PRKCB/PPP3CA	4
hsa05120	Epithelial cell signaling in Helicobacter pylori infection	3/54	70/8016	0.01151062	0.025102948	0.010182967	JUN/CASP3/CXCL2	3
hsa04270	Vascular smooth muscle contraction	4/54	132/8016	0.011770178	0.025398806	0.010302982	ADRA1D/PRKCA/PRKCB/CALM1	4
hsa03320	PPAR signaling pathway	3/54	76/8016	0.014370984	0.030688039	0.01244855	RXRA/PPARG/MMP1	3
hsa05204	Chemical carcinogenesis	3/54	82/8016	0.017600508	0.03719695	0.015088878	PTGS2/ADH1C/CYP1B1	3
hsa04911	Insulin secretion	3/54	86/8016	0.019960958	0.041668682	0.016902829	CHRM3/PRKCA/PRKCB	3
hsa04934	Cushing syndrome	4/54	155/8016	0.020122924	0.041668682	0.016902829	AHR/E2F1/E2F2/CDK2	4
hsa04540	Gap junction	3/54	88/8016	0.021203742	0.043467672	0.017632586	PRKCA/CDK1/PRKCB	3
hsa04310	Wnt signaling pathway	4/54	160/8016	0.022321682	0.045306384	0.018378456	JUN/PRKCA/PRKCB/PPP3CA	4
hsa04630	JAK-STAT signaling pathway	4/54	162/8016	0.023240916	0.046709685	0.018947703	BCL2/IL-6/STAT1/IL-4	4
hsa00350	Tyrosine metabolism	2/54	36/8016	0.024244872	0.048254357	0.019574296	ADH1C/MAOB	2

## Data Availability

The article deals with the establishment of the TCMSP database. The authors did not get permission to share the data.

## Supplementary Materials

Supplementary Materials Supplementary materials include Supplementary Table 1, Table 2, Table 3, and Table 4. Table 1: molecular function of GO enrichment of putative ZLJSD targets with BLCA. Table 2: cell component of GO enrichment of putative ZLJSD targets with BLCA. Table 3: KEGG enrichment of putative ZLJSD targets with BLCA. Table 4: another version of KEGG enrichment of putative ZLJSD targets with BLCA.
